# Experimental Analysis of the Effect of Rehabilitation Intervention on Tennis Players by Joint Injury Treatment

**DOI:** 10.1155/2022/4625719

**Published:** 2022-06-21

**Authors:** Ligang Ma, Xuedou Yu, Ruihua He, Yakun Gao, Xiaoliang Li

**Affiliations:** ^1^Hebei University of Engineering, Handan, 056038 Heibei, China; ^2^Capital University of Physical Education and Sports, Beijing 100191, China

## Abstract

In the process of competition and training, tennis players often carry out explosive force and extreme centripetal and eccentric contraction, while the ligament and joint capsule on the shoulder joint are relatively weak, which also makes the joint often appear injury caused by overuse. It has been the direction of scientific research to help athletes recover their functions and return to the arena through effective rehabilitation training and prerehabilitation training. In this paper, the reliability and short-term effect of wearing dynamic and static shoulder joint brace after arthroscopic repair of rotator cuff injury were studied through a controlled trial of tennis exercise for the treatment of shoulder injury. The purpose of this study was to apply the dynamic and static shoulder joint brace to patients with rotator cuff injury and shorten the recovery time of shoulder joint function the operation. This paper also studies the therapeutic effect verification of patients with rotator cuff injury during rehabilitation period by wearing shoulder joint brace with dynamic and static combination. Through the comparison between the experimental group and the control group, it is verified that the effect of rehabilitation intervention is better than that of the control group, which shows that the use of dynamic and static shoulder joint brace can improve the range of motion of shoulder joint and patient satisfaction, and the effect increases with time. This study improves the shoulder strength of tennis players through functional training, demonstrates the value and significance of functional training for the development of tennis through experiments, and provides a reference for athletes to improve their physical fitness training. At the same time, the research content of this paper can also provide references and promotion for sports events.

## 1. Introduction

Tennis is one of the most professional sports in the world. Every year, different levels of competitions are held all over the world. The most fascinating thing about tennis is the game between the opponents in all aspects. The length of each point, the choice of shot, the strategy, the duration of the game, the weather, and the opponent all affect the player's performance [1]. In a tennis match, players need to make hundreds of sudden stops and turns, in which quick start and change of direction are the basis of tennis movement. Since there is no time limit on the game, this can result in games lasting less than an hour or up to three hours. The uncertainty of competition duration requires tennis players to have a better level of anaerobic training to improve their performance in sports competitions [2].

Athletes need to have good specific physical abilities such as strength, speed, agility, endurance, and flexibility. In the fierce competition, due to the sports characteristics of tennis, it is necessary to have the good physical fitness to cope with the high-intensity and long-term competition and the positive and effective recovery after the match [3]. On the contrary, it may lead to certain sports injuries for athletes. Active rehabilitation training can enable athletes to return to the arena as soon as possible and achieve better results. Prerehabilitation is a training method adopted before the injury, which can help athletes effectively control injuries. In recent years, it is often used in the physical training of athletes with a high risk of injury [4]. Professional tennis players generally have at least one kind of injury, which will not only directly affect the performance of sports but also affect the effect of daily training. Active rehabilitation after injury and effective prerehabilitation before an injury can solve the plight of some tennis players, so it is very necessary to study the rehabilitation and prerehabilitation of tennis players [5].

The shoulder joint is a common injury site for tennis players. As one of the joints with the largest range of motion in the human body, it can move in a wide range of anatomical structures. The humeral head of the shoulder joint is large and spherical, the glenoid is shallow and small, only surrounding 1/3 of the humeral head, and the joint capsule is thin and loose [6]. Although the structural characteristics of the shoulder joint ensure its flexibility, its stability is also reduced. It is one of the most unstable joints in the whole body, which also determines the low flexibility and stability of the shoulder joint of athletes. More and more studies have shown that shoulder injuries are related to shoulder instability and scapular motion trajectory [7]. In such movements as overhead, such as the service link of athletes, repeated shoulder joint adduction and internal rotation will increase the risk of shoulder joint injury. The causes of most shoulder injuries of tennis players can be found in anatomy, physiology, and biomechanics. Shoulder joint injuries are often combined in various ways, resulting in specific injury patterns and dysfunction, so it is very important to understand the possible changes in shoulder joint in advance and feasible targeted rehabilitation programs for shoulder joint rehabilitation. Tennis players will inevitably suffer from various shoulder injuries in training or on the court. It has been the direction of scientific research to help athletes recover their functions and return to the court through effective rehabilitation training and prerehabilitation training. At present, after the shoulder joint is injured, local pain management, muscle release, joint loosening, and other methods are usually carried out first to help restore the basic functional state of the shoulder joint. Recovery and regeneration after exercise is also an important part. Stretching and other methods can help the shoulder muscles and the surrounding joint capsule to increase their mobility, which is conducive to the rehabilitation of shoulder injury [8].

Winge prospectively recorded injuries in 104 randomly selected elite tennis players during the 1984 outdoor tennis season and found that upper limb injuries were the most common and shoulder injuries were the most common among upper limb injuries [9]. It also pointed out that arm and shoulder injuries are more common in tennis than in badminton and squash, which may be caused by heavier tennis rackets. Tennis players constantly repeat forehand, backhand, serve, and other movements in their daily training. These movements are easy to cause tension in shoulder joint internal rotation and adductor muscles. If the related muscles are not released in time, acromion impact will easily occur, leading to movement deformation or aggravation of symptoms. However, this can improve the health of the shoulder joint by increasing strength, endurance, and flexibility training at the same time as technical training [10]. Teacher Ji Junfeng found that shoulder joint injury was the most common, more than 70%, followed by waist and knee [11].

In this study, functional strength training is an innovation of current physical training, which is based on the optimization and progress, focusing on the application of training benefits to tennis skills.

Through the reference and collection of functional training concepts, this study screened functional training methods under the guidance of experts and then formulated individualized training programs according to the actual situation of tennis players. It is conducive to more coordinated batting action, strengthening the working efficiency of shoulder joint power chain, making the power transmission from bottom to top more smoothly, improving the level of physical training of athletes, and reducing the risk of sports injury.

The main innovations of this paper are the following:

1. This paper analyzes the late restorative rehabilitation treatment of shoulder joint injury of tennis players and uses functional strength training to intervene and improve the athletes' physical function
2. For the recovery of joint movement in rehabilitation treatment, the use of dynamic and static shoulder joint braces to provide protection for athletes' shoulder joints and reduce the risk of injury caused by injury rehabilitation

## 2. Analysis of Shoulder Joint Injury in Tennis

In modern tennis, forehand and serve account for more than 75% of the points. S. Koviks found that the concentric contraction of the shoulder joint in the horizontal plane is the contraction of the middle deltoid, posterior deltoid, latissimus dorsi, infraspinatus, teres minor, and wrist extensor muscles. The eccentric contraction is by the anterior deltoid, pectoralis major, and subscapularis [12]. During acceleration, the latissimus dorsi, anterior deltoid, subscapularis, biceps brachii, and pectoralis major muscles all move the racquet in the direction of the ball in a concentric contraction. In the swing phase after hitting the ball, the movement of the shoulder joint is completed by the eccentric contraction of infraspinatus, teres minor, posterior deltoid, rhomboid, serratus anterior, trapezius, triceps brachii, and extensor muscle group [13]. The two-handed backhand uses many of the same muscles as the forehand but requires more trunk rotation, and the power of the two-handed backhand lies in the non-dominant arm and wrist. The action of serving can be divided into three stages: accumulation, acceleration, and following the ball. In the accumulation (preparation) stage, the body will accumulate energy. In the acceleration stage, the power will be released after contact with the ball. The final period with the ball (deceleration) requires a strong centrifugal force to help the upper and lower body decelerate [14].

There is an imbalance between the muscles of the posterior rotator cuff (external rotation) and the internal rotator cuff (internal rotation) of professional athletes. The internal rotator is more numerous and powerful than the external rotator. The internal rotator can produce 1.75 times as much isometric torque as the external rotator. This imbalance makes the external rotator more vulnerable to injury to the main internal and external rotators, as shown in Figure 1.

Through repeated shoulder isokinetic tests, it was found that the internal rotation muscle strength of the athlete's dominant arm increased by 15-30% compared with that of the non-dominant arm. When the external rotation muscle strength of the athlete's dominant arm remained unchanged or decreased, the greater the internal rotation muscle strength, the greater the imbalance between the external and internal rotation muscles [15].

It is found that the muscle strength and endurance of the rotating muscle group have a decisive impact on the action technology of tennis players. Whether serving or playing for a long time, the rotating muscle group is indispensable. A strong shoulder will help to store energy for release during the forehand stroke, and it is important to have enough muscle strength to effectively decelerate the arm during the swing after the stroke to prevent shoulder and arm injuries [16]. Tennis matches frequently use serve and forehand to hit the ball. The shoulder joint on this site is easy to cause fatigue and even injury due to loss of dynamic stability. Therefore, in the training plan, we should strengthen the balance of internal and external rotation muscles, scapular stability, rotation muscles, and other training according to the design method of tennis special sports [17].

## 3. Study on Clinical Diagnostic Criteria

### 3.1. TCM Diagnostic Criteria

Refer to the industry standard of traditional Chinese medicine of the People's Republic of China, Criteria for Diagnosis and Efficacy of TCM Diseases (ZY/T001.9-94).

1. Clinical expression: shoulder joint is aching; there is pain in the triangle area, which is more severe at night. Or there is limitation of movement, active flexion or abduction of the shoulder, with a history of old shoulder axis injury.
2. Physical examination: tenderness under the acromion or at the greater tuberosity of the humerus or positive drop arm test and impact test, pain arc: recovery of abduction 60-120 degrees, and glenohumeral snap or friction sound. Muscle atrophy or joint contracture may occur in patients with a course of more than 3 months
3. Auxiliary examination: X-ray examination: shoulder joint plain film; the bone may have hyperosteogeny or no obvious abnormalities; ultrasonography showed that there was echo enhancement disorder in the rotator cuff, low echo or high and low mixed echo lesions, and effusion in the rotator cuff area. Magnetic resonance imaging (MRI): the rotator cuff tissue is damaged but not completely torn [18]

### 3.2. Diagnostic Criteria of Western Medicine

1. Shoulder pain or muscle weakness, the intermittent onset of pain, aggravated at night, and pain in front of the shoulder joint and anterolateral
2. Overhead pain, weakness, limitation of active movement, and tenderness at the large tubercle in front of the shoulder
3. Physical examination: pain arc sign and impact test were positive, and abdominal pressure test or lift-off test was positive
4. Imaging examination: X-ray examination: the bony structure of the shoulder joint and the shape of the acromion were judged. In some cases, there was obvious local hyperosteogeny

Magnetic resonance imaging (MRI) can determine the location of rotator cuff injury and the severity of the tear, which is of high value in the diagnosis of the disease [19].

## 4. Research Methods

### 4.1. Grouping Method

According to the sample size estimation formula in clinical research methodology of combined use of traditional Chinese medicine and Western medicine [20],

(1) $$\begin{array}{c} n_{1}=n_{2}=\frac{2\left[{\left(u_{a}+u_{\beta }\right)}^{2}o^{2}\right]}{\lambda^{2}}. \end{array}$$

According to the literature [21], the ASES score of the ordinary shoulder joint brace group was 76.68 ± 10.49, and the ASES score of the shoulder joint abduction brace group under the guidance of dynamic and static combination was 85.75 ± 9.07. *μ*_*α*_ = 1.96, *μ*_*β*_ = 1.28, *α* = 0.05, and *β* = 0.10 were taken. According to PASS15 software, 26 cases were needed in each group. Considering the loss and loss of follow-up, the maximum loss rate of 15% was taken. There were about 30 cases in each group.

### 4.2. Treatment Method

Patients in the control group wore the conventional shoulder abduction brace and received rehabilitation exercise after shoulder arthroscopy, and the conventional shoulder abduction brace was removed during functional exercise.

Patients in the experimental group were given a portable three-dimensional scanner to obtain the three-dimensional scanning data of the affected upper limb and lateral chest wall before operation. After obtaining the data, the 3D shoulder joint brace was designed and printed. The brace includes the movable shoulder joint and elbow joint, which conforms to the principle of dynamic and static combination of orthopedics and traumatology of traditional Chinese medicine, as shown in Figure 2.

After arthroscopic shoulder surgery, the patients wore a dynamic and static shoulder joint brace and received rehabilitation exercises. Patients can wear the shoulder joint brace with functional exercises, and surgeons can adjust the range of motion of the shoulder joint brace according to the location of rotator cuff injury to limit the direction of shoulder joint motion that affects rotator cuff repair and retain the rest direction of shoulder joint motion.

### 4.3. Comparison of Course of Disease

The course data of the two groups did not conform to the normality distribution (Shapiro‐Wilk = 0.623, 0.655, *P* = 0.000, 0.000 < 0.01) by the normality test; there was no significant difference between the two groups by the independent sample Mann-Whitney *U* test (Mann‐Whitney *U* = 389.500, *P* = 0.368 > 0.05), as shown in Table 1.

### 4.4. Normality Test of VAS Recovery Score Comparison between the Two Groups

The VAS recovery score data of the experimental group and the control group before surgery (Shapiro‐Wilk = 0.898, 0.889, *P* = 0.007, 0.005 < 0.01), 6 weeks after surgery (Shapiro‐Wilk = 0.860, 0.860, *P* = 0.001, 0.001 < 0.01), and 12 weeks after surgery (Shapiro‐Wilk = 0.799, 0.799, *P* = 0.000, 0.000 < 0.01) did not conform to normal distribution, so the nonparametric rank sum test was used.

By Mann-Whitney *U* test, there was no significant difference in VAS score between the two groups before operation (Mann‐Whitney *U* = 459.500, *P* = 0.886 > 0.05), and there was no significant difference in VAS score between the two groups 6 weeks after operation (Mann‐Whitney *U* = 450.500, *P* = 1.000 > 0.05). There was no significant difference in VAS score between the two groups at 12 weeks after operation (Mann‐Whitney *U* = 450.500, *P* = 1.000 > 0.05).

Intragroup comparison: there was significant difference in VAS scores between the two groups by Friedman test (Friedman = 58.513, 59.000; *P* = 0.000, 0.000 < 0.01). Using the Wilcoxon *Z* test, there was a significant difference in VAS scores between 6 weeks after surgery and before surgery in the experimental group (Wilcoxon *Z* = −4.563, *P* = 0.000 < 0.01), between 12 weeks after surgery and before surgery (Wilcoxon *Z* = −4.798, *P* = 0.000 < 0.01), and between 12 weeks and 6 weeks after surgery. There was significant difference in VAS recovery score (Wilcoxon *Z* = −4.764, *P* = 0.000 < 0.05).

In the control group, there was a significant difference in the VAS score at 6 weeks after operation compared with that before operation (Wilcoxon*Z* = −4.729, *P* = 0.000 < 0.01), at 12 weeks after operation compared with that before operation (Wilcoxon *Z* = −4.796, *P* = 0.000 < 0.01), and there was a significant difference in the VAS recovery score at 12 weeks compared with that at 6 weeks after operation (Wilcoxon *Z* = −4.846, *P* = 0.000 < 0.01).

## 5. Experimental Analysis

### 5.1. Experimental Data

The design of this experiment is mainly based on the “Sports Injury” and “Sports Rehabilitation Treatment,” with a view to the empirical study of functional stretching rehabilitation on the shoulder complex stretching of tennis players [22]. Through the combined domestic core journals, master's papers, and American functional advocates, the functional rehabilitation cycle in China is generally 6 to 12 weeks. This rehabilitation is a local stretching rehabilitation with shoulder complex as the core, so the rehabilitation cycle is set at 8 weeks. And the rehabilitation content is based on the specific implementation methods of functional rehabilitation expert Mike Boyle and the American Physical Fitness Association (NSCA) [23].

Based on this, a preexperiment will be conducted on the subjects before the experiment, and the test indicators, rehabilitation methods, and rehabilitation load of this experiment will be evaluated. The inappropriate test indicators and methods should be adjusted and improved in time. The experimental conditions were strictly controlled during the experiment to ensure the effectiveness of the experimental process. After the experiment, the two groups of subjects were tested again, and statistical analysis was carried out to explore the effect of functional stretching rehabilitation.

### 5.2. Experimental Method

The two groups of athletes will carry out shoulder stretching rehabilitation after each routine rehabilitation, each time for about 30 minutes. Because the local rehabilitation of the upper body is the main part, the control of the rehabilitation intensity is basically 50-70% of HRmax, which ensures that the rehabilitation intensity of the two groups tends to be consistent [24].

The experimental group was designed with the method of functional rehabilitation combined with the special action mode of tennis. The rehabilitation process is shown in Table 2.

### 5.3. A Comparative Analysis of the Test Results of the Experimental Group and the Control Group before the Experiment

Before the experiment, the shoulder joint recovery test, in situ tennis throwing, and other related indicators of the experimental group and the control group were tested, and the test data are shown in Tables 3 and 4.

The comparison of data before the experiment is shown in Figure 3.

Shoulder joint stability tests of the members of the experimental group and the control group before the experiment are shown in Table 5.

In Table 5, before the experiment, there was no significant difference between the experimental group and the control group in the test results of shoulder joint stability, tennis throw, medicine ball throw with both hands, holding racket hand throw, and nonholding racket hand throw (*P* > 0.1). In addition, there was no significant difference in age, height, weight, rehabilitation years, and other related information (*P* > 0.1), indicating that the experimental grouping was reasonable.

### 5.4. Comparative Analysis of the Test Results between the Experimental Group and the Control Group after the Experiment

#### 5.4.1. Test Results of the Experimental Group and the Control Group after the Experiment

After 8 weeks, the subjects were tested for shoulder joint recovery test, tennis throw, two-handed head forward throw of medicine ball, and other related indicators. The test results are shown in Tables 6 and 7.

After the experiment, the test results were compared and analyzed. The independent sample *t*-test was carried out on the relevant indicators of functional rehabilitation and traditional stretching rehabilitation of shoulder joint complex in Tables 6 and 7. The test results are shown in Table 8.

In Table 8, after 8 weeks of experiment, there is no significant difference between the experimental group and the control group in tennis throwing, holding racket throwing, and nonholding racket throwing (*P* > 0.1), but there is significant difference in shoulder joint recovery test and two-handed head forward throwing medicine ball test (*P* < 0.1).

#### 5.4.2. Comparison and Analysis of Test Index Changes between Experimental Group and Control Group after Experiment

After the experiment, the index change values of the test items in the experimental group and the control group were counted, and the statistical results are shown in Tables 9 and 10.

After the experiment, independent sample *t*-test and statistical analysis were performed on the change values of the two groups of test indicators, as shown in Table 11.

The analysis of the test indexes of the experimental group and the control group is shown in Figure 4.

According to the data in Table 11 and Figure 4, the shoulder joint recovery of the experimental group increased by 15.2% and that of the control group increased by 5.2%. Compared with before the experiment, the average increase of throwing the medicine ball with both hands was 15.18%, and the control group increased by 1.2%. The data of increasing value in Tables 9 and 10 were tested by independent sample *t*-test to obtain the two groups of test indicators *P* < 0.1, indicating that there was a significant difference between the experimental group and the control group after the experiment. The data of the added values in the table were tested by the independent sample *t*-test, and the data showed *P* > 0.1, indicating that there was no significant difference between the two groups of testers.

After 8 weeks of the experiment, the shoulder joint recovery of the testers in the experimental group and the related indexes reflecting the stretching of the shoulder joint complex was improved, except for throwing a medicine ball without holding the racket in situ. *P* was less than 0.1, showing significant differences. In the control group, *P* was less than 0.1, and the percentage of muscle strength increase of nonholding hands was better than that of the experimental group, indicating that functional stretching rehabilitation can effectively improve the recovery of the shoulder complex, and both traditional stretching rehabilitation and functional rehabilitation can improve shoulder muscle strength. Traditional stretching rehabilitation is more effective in improving the muscle strength of the weak shoulder complex.

## 6. Conclusion

This study improves the shoulder strength of tennis players through functional training, demonstrates the value and significance of functional training in the development of tennis through experiments, and provides a reference for coaches and athletes to improve tennis physical training.

The main contents are the following:

1. Prerehabilitation training intervention can maintain the functional status of shoulder joint and improve the coordination of intermuscular force. Prerehabilitation can improve the level of shoulder muscle strength and improve the ability of antagonistic muscle to work
2. In rehabilitation training, the speed of muscle contraction is related to the length of muscle. Increasing muscle elasticity and stretching muscle in training are helpful to the development of contraction speed

Comparative analysis before and after intervention showed that muscle strength changed greatly in high-speed (180°/s) exercise. In the case of wearing a dynamic and static shoulder joint brace, muscle release, stretching, and exercise intervention can effectively improve the flexor and extensor strength of shoulder joint in high-speed movement.

In future work, the digital stadium and digital-physical training equipment will be “networked.” Digital monitoring is mainly used to monitor the changes in athletes' muscle strength, nerve response, and other training conditions. For physical fitness digital equipment, it is necessary to purchase some relevant digital training systems according to the situation for athletes' multidimensional training.

## Figures and Tables

**Figure 1:** Internal rotators vulnerable to tennis.

**Figure 2:** 3D shoulder brace.

**Figure 3:** Comparison of data before experiment.

**Figure 4:** Analysis of test indexes.

**Table 1:** Comparison of disease course between the two groups.

Groups	Course of disease (month)
Experimental group	30.67 (1.00, 3.00, 6.00)
Control group	27.25 (1.00, 1.50, 2.00)

**Table 2:** Comparison of rehabilitation process.

	Traditional stretching rehabilitation implementation process	Functional extension rehabilitation implementation process
Rehabilitation goals	1. Strengthens the muscular extension of the shoulder complex	Improve the shoulder complex muscle stretching of tennis players, and combine the rehabilitation benefit of functional stretching with tennis specialty
	2. Strengthen the athletes' consciousness of stretching and rehabilitation to reduce the loss	
Rehabilitation task	Cooperate with the tennis project and choose the corresponding stretching rehabilitation action	Combined with the specific movement pattern of tennis, the corresponding functional stretching rehabilitation is designed to improve specific skills
Rehabilitation principle	Increases neuromuscular excitability and the cross-sectional area of muscle fibers. Work the big muscles first and then work the small muscles	Push and pull exercises in the horizontal direction and those in the non-horizontal direction in appropriate proportions. For each set of pushing exercises, there should be at least one set of pulling exercises [25]

**Table 3:** Statistical table of test results of the experimental group before the experiment.

User	Scapular stability	Tennis far away (M)	Two hands on your hands and throw a solid ball (m)	Holding hands in place (m)	Nonclapped hands and throw away (m)
A1	9.3	15.2	10.6	13.2	12.1
A2	8.6	17.3	9.8	13.7	11.5
A3	8.9	16.8	11.5	12.9	11.9
A4	9.2	16.9	10.4	13.5	11.4
A5	9.5	17.2	10.7	13.6	11.3
Average	9.1	16.68	10.6	13.38	11.64
Standard deviation	0.75	0.64	0.77	0.85	0.91

**Table 4:** Statistical table of test results of the control group before the experiment.

User	Scapular stability	Tennis far away (M)	Two hands on your hands and throw a solid ball (m)	Holding hands in place (m)	Nonclapped hands and throw away (m)
A1	8.3	9.3	10.2	11.0	12.0
A2	8.1	9.5	11.6	11.2	11.7
A3	8.2	9.7	11.7	11.2	11.3
A4	8.1	10.0	11.6	10.9	11.2
A5	8.0	9.8	10.9	10.9	11.2
Average	8.1	9.7	11.2	11.1	11.5
Standard deviation	0.45	0.37	0.41	0.68	0.93

**Table 5:** Comparative analysis of test results between the experimental group and the control group before the experiment.

Test project	Experimental group (*x* ± *s*)	Control group (*x* ± *s*)	*P*
Shoulder joint recovery	9.1 ± 0.75	8.56 ± 0.45	0.82 > 0.1
Tennis throw away	16.68 ± 0.64	9.08 ± 0.37	0.43 > 0.1
Throw the medicine ball forward with both hands	10.6 ± 0.77	1018 ± 0.41	0.67 > 0.1
Hold the racket in place and throw it far	13.38 ± 0.85	13.16 ± 0.68	0.97>0.1
Throw far without holding the racket in place	11.64 ± 0.91	9.66 ± 0.93	0.93>0.1

**Table 6:** Statistical table of test results of the experimental group after the experiment.

Name	Shoulder joint recovery	Tennis throw away (m)	Throw the medicine ball forward with both hands (m)	Hold the racket in place and throw it far (m)	Throw far without holding the racket in place (m)
A1	10.6	15.5	11.1	14.2	13.2
A2	9.3	17.7	10.7	14.6	12.5
A3	9.9	17.4	12.4	13.9	12.8
A4	10.5	17.7	11.6	14.3	12.1
A5	10.9	17.9	11.7	14.4	12.1
Average number	10.24	17.24	11.5	14.28	12.54
Standard deviation	0.53	0.17	0.53	0.89	0.96

**Table 7:** Test results of the control group after the experiment.

Name	Shoulder joint recovery	Tennis throw away (m)	Throw the medicine ball forward with both hands. (m)	Hold the racket in place and throw it far (m)	Throw far without holding the racket in place (m)
A1	8.5	9.6	9.9	12.8	11.9
A2	8.7	9.2	10.3	13.7	12.3
A3	8.2	8.7	10.7	13.6	12.4
A4	8.1	9.3	9.8	12.9	11.5
A5	9.3	8.6	10.2	12.8	11.7
Average number	8.56	9.08	10.18	13.16	9.66
Standard deviation	0.22	0.41	0.99	0.86	0.99

**Table 8:** Comparative analysis of test results between experimental group and control group after the experiment.

Test items	Experimental group	Control group	*P*
Shoulder joint recovery	9.24 ± 0.53	8.17 ± 0.22	0.071 < 0.1
Tennis throw away (m)	11.05 ± 0.17	9.72 ± 0.41	0.36 > 0.1
Throw the medicine ball forward with both hands (m)	12.36 ± 0.53	11.24 ± 0.99	0.072 < 0.1
Hold the racket in place and throw it far (m)	13.23 ± 0.89	11.11 ± 0.86	0.83 > 0.1
Throw far without holding the racket in place (m)	13.41 ± 0.96	11.51 ± 0.99	0.81 > 0.1

**Table 9:** Changes of test indexes in the experimental group after the experiment.

Name	Shoulder joint recovery	Tennis throw away (m)	Throw the medicine ball forward with both hands. (m)	Hold the racket in place and throw it far (m)	Throw far without holding the racket in place (m)
A1	1.31	0.33	0.58	1.02	1.15
A2	0.72	0.27	0.93	0.97	1.09
A3	0.96	0.29	0.95	1.09	0.93
A4	1.27	0.31	1.21	0.89	0.78
A5	1.43	0.34	1.09	0.87	0.81
Average number	1.14	0.31	0.95	0.97	0.95

**Table 10:** Changes of test indexes in the control group after the experiment.

Name	Shoulder joint recovery	Tennis throw away (m)	Throw the medicine ball forward with both hands. (m)	Hold the racket in place and throw it far (m)	Throw far without holding the racket in place (m)
A1	0.2	0.3	-0.3	1.8	-0.1
A2	0.6	-0.3	-1.3	2.5	0.6
A3	0	-1	-1	2.4	1.1
A4	0	-0.7	-1.8	2	0.3
A5	1.3	-1.2	-0.7	1.9	0.5
Average number	0.42	-0.38	-1.02	2.12	0.48

**Table 11:** Comparison and analysis of change values of test indexes between the experimental group and the control group after the experiment.

Test index	Amplitude of increase in experimental group (%)	Amplitude of increase in control group (%)
Shoulder joint recovery	15.2%	5.4%
Tennis throw away (m)	3.9%	2.3%
Throw the medicine ball forward with both hands (m)	15.18%	1.2%
Hold the racket in place and throw it far (m)	7.3%	2.6%
Throw far without holding the racket in place (m)	6.5%	5.5%

## Data Availability

The data used to support the findings of this study are available from the corresponding author upon request.
